# BERT-PPII: The Polyproline Type II Helix Structure Prediction Model Based on BERT and Multichannel CNN

**DOI:** 10.1155/2022/9015123

**Published:** 2022-08-24

**Authors:** Chuang Feng, Zhen Wang, Guokun Li, Xiaohan Yang, Nannan Wu, Lei Wang

**Affiliations:** ^1^School of Computer Science and Technology, Shandong University of Technology, Zibo 255000, China; ^2^Key Laboratory of Symbolic Computation and Knowledge Engineering of Ministry of Education, Jilin University, Changchun 130012, China

## Abstract

Predicting the polyproline type II (PPII) helix structure is crucial important in many research areas, such as the protein folding mechanisms, the drug targets, and the protein functions. However, many existing PPII helix prediction algorithms encode the protein sequence information in a single way, which causes the insufficient learning of protein sequence feature information. To improve the protein sequence encoding performance, this paper proposes a BERT-based PPII helix structure prediction algorithm (BERT-PPII), which learns the protein sequence information based on the BERT model. The BERT model's *CLS* vector can fairly fuse sample's each amino acid residue information. Thus, we utilize the *CLS* vector as the global feature to represent the sample's global contextual information. As the interactions among the protein chains' local amino acid residues have an important influence on the formation of PPII helix, we utilize the CNN to extract local amino acid residues' features which can further enhance the information expression of protein sequence samples. In this paper, we fuse the *CLS* vectors with CNN local features to improve the performance of predicting PPII structure. Compared to the state-of-the-art PPIIPRED method, the experimental results on the unbalanced dataset show that the proposed method improves the accuracy value by 1% on the strict dataset and 2% on the less strict dataset. Correspondingly, the results on the balanced dataset show that the AUCs of the proposed method are 0.826 on the strict dataset and 0.785 on less strict datasets, respectively. For the independent test set, the proposed method has the AUC value of 0.827 on the strict dataset and 0.783 on the less strict dataset. The above experimental results have proved that the proposed BERT-PPII method can achieve a superior performance of predicting the PPII helix.

## 1. Introduction

Cowan et al. firstly discovered a special protein secondary structure the polyproline II (PPII) helix [1] which differs from the conventional protein secondary structure such as *α*-helix, *β*-pleated sheet, and random coil. The PPII helix consists of almost 3~8 amino acid residues, and it occupies only about 2% in the protein. The PPII helix has special biological characteristics and plays a crucial role in biochemical fields such as signal transduction, cell movement, and immune response [2, 3]. There are many interactions between the PPII helix and proteins or nucleic acids, such as SH3, WW, EVH1, GYF, UEV, and inhibitor proteins, which interact with the PPII helix [4–6]. Meanwhile, the PPII helix relates to many difficult diseases, such as the Alzheimer's disease and Parkinson's disease [7, 8]. Thus, it is very important to correctly predict the PPII helix. At present, the prediction of conventional secondary structures has made great achievements. But, a few researchers focused on the prediction of PPII helix. Furthermore, the PPII helix is very rare, which makes it become difficult to predict the PPII helix.

Anfinasen et al. [9] proposed the famous conclusion that protein sequence determines its spatial structure on the basis of experiments in 1961. Similarly, PPII structure is the same. The protein structure determination methods can be divided into two categories: traditional research methods of protein structure analysis and computational biology prediction methods. The traditional research methods use the X-ray crystal diffraction technology and the nuclear magnetic resonance imaging technology to predict the protein structure. It is hard for human to recognize, and the determination time is long. To solve the above problem, researchers proposed to predict PPII helices using protein sequence data in the bioinformatics field. However, the sequence based prediction models manually extract the features, and it usually leads to an inferior prediction result. Fortunately, the deep learning networks have powerful built-in feature extractors and have been widely used to extract protein feature information [10–12].

Recently, the researchers proposed to further improve the proteins features by using the natural language processing (NLP) technology. Proteins and languages are similar in concept [13], and Ofer et al. have descripted the relationship among the natural language processing, machine learning, and protein sequences. Ofer considers the protein sequence as an unknown language. Correspondingly, the amino acid is a word in biological vocabulary, and the biological sequence (such as DNA sequence and protein sequence) is text information. More and more natural language processing (NLP) techniques have been applied to solve the sequence prediction problems in bioinformatics [14–17].

The Bidirectional Encoder Representation from Transformers (BERT) [18] is a simple but powerful language model. We can pretrain BERT with the natural language corpus and use the trained BERT to transfer learning the biological sequences. Ho et al. [19] proposed the FAD-BERT model to predict the flavin adenine dinucleotide (FAD) binding sites, which can overcome the problem of insufficient feature learning caused by the shortage of training data. Charoenkwan et al. [20] used BERT4Bitter model to predict bitter peptides without system designing and feature coding selection. BERT4Bitter model automatically generate feature descriptors based on the original protein sequence. Li et al. [21] used the pretrained BERT model to learn both the protein sequence features and the amino acid hydrophilic features. As a result, it can improve the performance of predicting the missense mutations in protein sequences. To improve the encoding performance, Ali Shah et al. [22] utilized the pretrained BERT language model to extract the protein sequences features, which can effectively distinguish the three kinds of glucose transporter families. Le et al. [23] regarded DNA sequence as a natural language sentence and used BERT model to represent the DNA sequence information. It can capture the information which is equivalent to human language. BERT-m7G model [24] used the BERT model to convert RNA sequence information into feature matrix and select the optimal feature based on an elastic network. Finally, BERT-m7G model can effectively improve the prediction performance of RNA N7-methylguanosine.

As a special protein structure, many methods have been proposed to predict the PPII helix. Siermala et al. [25] firstly used the feed-forward neural network and back propagation algorithms to predict PPII helix structure. The prediction accuracy in reaches 75% on the datasets which has been eliminated more than 65% redundant sequences. Wang et al. [26] proposed to predict the PPII helix based on the support vector machine, and the prediction accuracy reached 70% on the dataset that further reduced homologous protein sequences. Lu et al. improved the artificial neural network [27] by jointly using the adjacent amino acid residue information and the one-hot encoding. Thus, Lu simultaneously use the improved artificial neural network, the support vector machine (SVM) [28], and the genetic neural network [29] to predict the PPII helix. O'Brien et al. [30] predict the PPII helix structure based on bidirectional recurrent neural network (BRNN). Its takes into account that the formation of PPII helix is affected by the remote residues, and other sequences are compared with the sequence to obtain a position-specific scoring matrix (PSSM) containing evolutionary information as a feature representation.

The existing PPII helix structure prediction methods usually adopt one kind of protein sequence code and only use the local or global protein sequence features. This will lead to an inferior performance. To solve the above problems, this paper uses the pretrained BERT model to improve the performance of protein sequences code. Each protein sequence is regarded as a sentence, and each amino acid is regarded as a word. This paper predicts the PPII helix structure by jointly using the local and global features. The flowchart of this algorithm is shown in Figure 1.

The proposed algorithm mainly includes three steps: learning global features, learning local features, and feature fusion.

(1) In the learning global features, we segment the protein amino acid sequences into many datasets with different sizes of sliding windows [34]. To further get the input of the BERT model, we separate each protein sequence sample into the amino acid residue by a space. After encoded by the BERT embedding layer, each amino acid residue is represented as a 768 dimensional context embedding vector. Then, each protein sequence sample is represented as *n* (*n* is window size) 768 dimensional vectors and 1 *CLS* vector. (2) In the learning local features, we use the multichannel CNN to extract n embedding vectors with 768 dimensions. The sizes of the multichannel CNN kernels are 3, 4, and 5, respectively. (3) In the feature fusion, we fuse the global *CLS* vector with the local features output by the multichannel CNN. Then, we use the softmax function to classify the fusion features.

In this paper, the BERT-PPII algorithm has the following innovations:

- The proposed method automatically extracts the feature extraction using protein primary sequences. This process has abandoned the system designing process and the feature selection procedure. Thus, it can avoid to manually extract the feature from raw amino acid sequences
- We use the pretrained BERT model to improve the protein sequence encoding, and features to enhance the ability of feature representation
- We design the comparative experiments on both the Strict_data dataset and the NonStrict_data dataset. The final experimental results show that the proposed BERT-based model is better than the existing algorithms

## 2. Materials and Methods

### 2.1. Problem Description

The PPII helix is a local spatial conformation between amino acid residues in the protein polypeptide chain. It usually consists of 3~8 amino acids. Its prediction task maps the protein sequence composed of 20 amino acids to the corresponding the PPII helix structure sequence. As shown in Figure 2, FQRP, the partial amino acid residues of protein sequence, is mapped to PPII helix structure. The existing PPII secondary structure prediction algorithms adopt only one kind of the protein encoding method, which causes the problem of insufficient learning features. The PPII helix is determined by both the local and the long-range among the amino acid residues in the protein chain. If the prediction process only uses local or global features, it will ignore the important PPII helix formation information and decrease the prediction accuracy.

To solve the problem of encoding protein sequence, this paper employs the BERT to improve the code of amino acids. Moreover, the *CLS* feature of the protein sequence obtained by BERT and the local feature of the protein sequence obtained by multichannel CNN are further integrated to effectively improve the expression ability of sample features. Our model mainly includes BERT embedding encoding and global feature extraction, local feature extraction by multichannel convolution, and multifeature fusion, which are described in Sections 2.2, 2.3, and 2.4, respectively.

### 2.2. Bert Embedding Encoding and Global Feature Extraction

More and more natural language processing (NLP) techniques have been employed to learn the feature descriptors of protein sequences, DNA sequences, and RNA sequences [14–17]. The BERT embedding layer can obtain semantic and syntactic information from the context of a sentence or paragraph, which enables to learn better features. Recently, most PPII helix structure prediction algorithms usually adopt only one kind of protein sequence feature encoding method. In order to learn the better features, the pretrained BERT model is used to improve the of the PPII helix structure prediction performance. We break this limitation by pretraining the model based on bidirectional encoder representation from transformers (BERT). The BERT model uses the multiattention mechanism to obtain the *CLS* feature vector. The *CLS* feature vector can fairly integrate the information of each amino acid residue in the sample. Finally, the *CLS* feature is considered as the global feature. The BERT model handles the migration task's input samples by the position encoding, self-attention mechanism, and residual connection.

Position encoding: Generally, the same characters with different locations are assigned the same feature description. Thus, they cannot capture the location information of the input text. To solve the above problem, the input samples are encoded according to the position of the character, as shown in Equation (1). *PE* denotes the position code of each input character. *pos* denotes the position of the character in the sequence. *dmodel* denotes the dimension of *WQ*(*x*). When the same characters appear in the input amino acid residues, they will have different feature codes obtained by the self-attentive mechanism due to the different position codes.

(1) $$\begin{array}{c} PE\left(pos,j\right)=\left\{\begin{array}{c} \sin\left(\frac{pos}{10000^{j}/d_{\text{model}}}\right),j=2i\\ \cos\left(\frac{pos}{10000^{j-1}/d_{\text{model}}}\right),j=2i+1 \end{array}\right.. \end{array}$$

After that, the protein sequence sample *X* = (*x*_1_, *x*_2_, *x*_3_, ⋯, *x*_n_) will be processed by word embedding query (*WQ*) and position coding (*PE*), as shown in Equation (2). *X*_input_ represents the input vector of BERT:

(2) $$\begin{array}{c} X_{\text{input}}=WQ\left(X\right)+PE. \end{array}$$

Self-attention mechanism: This paper utilizes the self-attention mechanism to capture the relationship among the amino acid residues of the input sample sequence, as shown in Equation (3). As a result, each character contains the information of the other characters, where *Q* = *X*_input_*W*^*Q*^, *K* = *X*_input_*W*^*K*^, *V* = *X*_input_*W*^*V*^. *Q*, *V*, and *K* are the query vector, value vector, and key vector, respectively. *W*^*Q*^, *W*^*K*^, and *W*^*V*^ are the weight matrices of *Q*, *K*, and *V*, respectively.

(3) $$\begin{array}{c} \text{Attention}\left(Q,K,V\right)=\text{softmax}\left(\frac{{QK}^{\text{T}}}{\sqrt{d_{k}}}\right)V. \end{array}$$

Residual connection: To avoid the problems of gradient disappearance and explosion during the training process, we establish the residual connection for the output of the self-attentive mechanism [36], as shown in Equation (4).

(4) $$\begin{array}{c} X_{\text{output}}=X_{\text{input}}+\text{Attention}\left(Q,K,V\right). \end{array}$$

During training the model, we normalize the data [37, 38] as shown in Equation (5). Thus, the algorithm can quickly and smoothly converge to the optimal solution. *μ* is the mean value of *X*_output_ and *σ* is the standard deviation of *X*_output_. When *σ* becomes 0, *ε* can avoid the denominator being 0. The training parameters *α* and *β* can compensate the information lost during the normalization process:

(5) $$\begin{array}{c} \text{LayerStandary}=\alpha \frac{X_{\text{output}}-\mu }{\sigma +\varepsilon }+\beta . \end{array}$$

To obtain the amino acid residues, we put the standardized features into the fully connected neural network followed by a residual connection and a standardization procedure.

To ensure the transformer's self-attention mechanism [39] has excellent representation ability, BERT model employs two pretraining tasks [18]: the “masked language model” (MLM) and the “next sentence prediction” (NSP). As a result, it can provide a better generalization result for the downstream tasks.

### 2.3. Local Feature Extraction by Multichannel Convolution

The interaction among the local amino acid residues in the protein chain has an important influence on the formation of the PPII helix. The protein sequences' features can be represented as matrices, and the local spatial correlations exist among the amino acids' features in the sequences. Moreover, the convolutional neural networks (CNNs) can handle the spatial correlation among the dense data in the network. In this paper, to obtain the relationships among the local amino acid residues, we further use the CNN to learn the feature of Bert's output vectors. The convolution neural networks capture the important local information of the protein sequence sample's features. Correspondingly, the pooling procedure learns the important local features. Thereafter, we obtain the final vector *η* by splicing the output vectors of the CNN layers.

In this paper, we design the CNN models with convolutional kernels of 3, 4, and 5, respectively (Section 3.5). As shown in Figure 3, the sample's local feature learning process mainly consists of the convolution operation and the pooling operation.

Convolution operation: We use the convolution operation to process the BERT layer's output matrix *B* = {*H*_1_, *H*_2_, ⋯*H*_n_}. Assuming the convolution kernel's size is *m*, each time the convolution is computed based on m word vectors. Generally, we slide the convolution kernel 1 step from top to bottom and divide *B* into {*H*_1:*m*_, *H*_2:*m*+1_, ⋯, *H*_*n*−*m*+1:*n*_}. Where *H*_*i*:*j*_ represents the concatenated vectors of {*H*_*i*_ ⋯ *H*_j_}. The vector *C* = {*c*_1_, *c*_2_, ⋯, *c*_*n*−*m*+1_} and the value *ci* is obtained by convolving *H*_*i*:*i*+*m*−1_, as shown in Equation (6):

(6) $$\begin{array}{c} c_{1}=W^{\text{T}}H_{i:i+m-1}+b. \end{array}$$

We initialize the convolution kernel's parameter (*W*) as a random uniform distribution. *b* is the bias variable.

Pooling operation: After the convolution operation, we perform a pooling operation on the text feature mapping vector *C* = {*c*_1_, *c*_2_, ⋯, *c*_*n*−*m*+1_}. For the results obtained with *q* convolution kernels, we use a global maximum pooling, as shown in Equation (7).

(7) $$\begin{array}{c} {\hat{C}}_{m}=\max\left(C_{m1},C_{m2},\cdots ,C_{mq}\right). \end{array}$$

We concentrate the features extracted with the kernel sizes *m* = (3, 4, 5) as the local feature vector *η*, as shown in Equation (8):

(8) $$\begin{array}{c} \eta =\left\{{\hat{C}}_{3},{\hat{C}}_{4},{\hat{C}}_{5}\right\}. \end{array}$$

### 2.4. Multifeature Fusion

A survey about the PPII helix structures prediction shows that most algorithms use the traditional features and manually select features to combine. Most research works only adopt the local features [26–29] or the global features [30–33], which decreases the accuracy of PPII helix structure prediction. Both the local and long-range interactions among amino acid residues determine the PPII helix. Therefore, the local features and global features are equally important in prediction the PPII helix. In this paper, we propose to fuse the protein sequences' local features *η* and the global features *CLS*, and the joint feature in Equation (9) is used to predict the PPII helix structure:

(9) $$\begin{array}{c} M=\text{concat}\left(CLS,\eta \right). \end{array}$$

The global feature *CLS* is obtained by the BERT model, and the local feature *η* is obtained by the multichannel CNN. We utilize the concat() algorithm to generate the final feature vector *M* = {*CLS*, *η*}. In this paper, we use the fusion feature *M* to predict the PPII helix structure.

## 3. Results and Discussion

### 3.1. Sample and Dataset

In this paper, we design the comparative experiments on the PPIIPRED dataset [30]. The filtering rules which define the PPII helix dataset [41] include two kinds of definitions: the “strict” and “less strict.” The filter criteria are percentage identity ≤30%, resolution ≤2.5, and *R*-value ≤0.25. The strict criteria include the trans filtering, the dihedral filtering, and the regularization filtering.

The trans filtering:

(10) $$\begin{array}{c} -145<\alpha C-70. \end{array}$$

The dihedral filtering:

(11) $$\begin{array}{c} -180<\Psi <-160, \end{array}$$

(12) $$\begin{array}{c} 90<\Psi <180, \end{array}$$

(13) $$\begin{array}{c} -105<\Phi <-45. \end{array}$$

The regularization filtering:

(14) $$\begin{array}{c} \frac{\sum_{k=1}^{n-1}d_{k,k+1}}{n}, \end{array}$$

(15) $$\begin{array}{c} d_{k-1,k}=\sqrt{{\left(\Psi_{i‐1}-\Psi_{i}\right)}^{2}+{\left(\Phi_{i}-\Phi_{i+1}\right)}^{2}}. \end{array}$$

Compared with the strict definition, the less strict definition removes the requirement: −105 < *Φ* < −45. Based on the above the definitions of the strict and less strict, we obtained the strict and less strict PPII helix structure datasets.

We used the sliding window technique [34] to select sequences as input samples. Assuming a protein sequence of length *L*, we can obtain 2 *m* + 1 protein sequence fragment to represent a single amino acid sample. So, the number of samples is *L*. Given the sliding window size is 13, the positive samples (PPII helix structure) and negative samples (non-PPII helix structure) are shown as in Figures 4(a) and 4(b).

For the problem of protein secondary structure identification, we predict the PPII helix based on sample center residues, since the prediction results relate to the information of the neighbor amino acid residues. The datasets processed by the sliding window are divided into training sets, validation sets, and test sets.  Table 1 is the dataset under strict definition (Strict_data), and Table 2 is the dataset under less strict definition (NonStrict_data).

To solve the serious imbalance problem between positive and negative samples, we employ the under-sampling method to randomly select the same number of negative samples as the positive samples in the original training data. We utilize both the negative samples and the positive samples as the training data. Furthermore, the training data is divided into training set and validation set, and their ratio is 4 : 1. The training set, the validation set, and the test set form a balanced dataset.

### 3.2. Analysis of Amino Acid Composition

We investigate the PPII helix structure and the non-PPII helix structure according to the relative frequency of the amino acid residues located in the center position of the PPII helix. In this study, the relative frequency of the various amino acids in the dataset is shown in Figure 5. It shows that A, E, L, and P are the amino acids in the PPII helical structure. A, G, L, and V are the main amino acids in the non-PPII helix structure. Compared with the non-PPII helix structure, amino acid P appears more frequently. Except the Proline (P), the other amino acids have no obvious characteristic in these two kinds of structure. The relative frequencies of the P in the middle of the PPII helix structure is about five times more than that in the middle of the non-PPII helix structure. Therefore, P can distinguish the PPII helix structure and the non-PPII helix structure effectively. Although P accounts for a large proportion, not all PPII helical structures contain P.

### 3.3. Evaluation Criteria

In this study, we adopt four commonly used metrics including sensitivity (Sens), specificity (Spec), accuracy (ACC) and Matthews correlation coefficient (MCC) to evaluate the performance. Their definitions are shown as follows:

(16) $$\begin{array}{c} Sensitivity=\frac{TP}{TP+FN}, \end{array}$$

(17) $$\begin{array}{c} Specificity=\frac{TN}{TN+FP}, \end{array}$$

(18) $$\begin{array}{c} Accuracy=\frac{TP+TN}{TP+FP+TN+FN}, \end{array}$$

(19) $$\begin{array}{c} MCC=\frac{TP*TN-FP*FN}{\sqrt{\left(TP+FP\right)\left(TP+FN\right)\left(TN+FP\right)\left(TN+FN\right)}}. \end{array}$$

Sensitivity represents the proportion of the positive samples which are correctly predicted. Specificity represents the proportion of the negative samples which are correctly predicted. ACC indicates the proportion of correctly classified samples; MCC represents the correlation coefficient between the observed category and the predicted binary classification. Its range is [−1,1]. We will get a better prediction result, when the MCC value is close to 1. TP represents the true positive. It is the number of positive samples correctly predicted. TF represents the true negative. It is the number of negative samples correctly predicted. FP represents the false positive. It is the number of negative samples incorrectly predicted. FN represents the false negative. It is the number of positive samples incorrectly predicted. AUC is the area under the ROC curve. We evaluate the generalization performance of the algorithm model based on AUC, and the value of a robust model is close to 1.

### 3.4. Optimal Sliding Window

To obtain the optimal window, we set up comparison experiments to measure the prediction performance with different windows. In this experiment, the step length is 2, and its value range is [11, 21]. The ROC of BERT-PPII model on the balanced Strict_data dataset and the NonStrict_data dataset is shown in Figures 6(a) and 6(b), respectively.  Figure 6(a) shows that the model has the best performance with the window size of [15, 17] and the AUC is 0.827.  Figure 6(b) shows that the model has the best performance with the window size of [13, 19] and the AUC is 0.783. Usually, the training time increases when the window size becomes. As a result, we set the window size as 15.

### 3.5. The Optimal Convolutional Kernel Combinations

To obtain the optimal channel number, we design the comparative methods combined with different *n*-gram channels as follows:

1. 3_kernel: contains 3-gram CNN channels
2. 3_4_kernel: a combination of 3-gram and 4-gram CNN channels
3. 3_4_5_kernel: a combination of 3-gram, 4-gram, and 5-gram CNN channels
4. 3_4_5_6_kernel: a combination of 3-gram, 4-gram, 5-gram, and 6-gram CNN channels
5. 3_4_5_6_7_kernel:a combination of 3-gram, 4-gram, 5-gram, 6-gram, and 7-gram CNN channels

We test these five methods on the balanced Strict_data dataset. The ROC curves are shown in Figure 7, and other performances are shown in Table 3. The experimental results show that the 3_4_5_kernel method has the best performance, in the range of [0.2,0.7] of FPR and the range of [0.7,1.0] of TPR, which is the most meaningful part for performance comparison. We use the 3_4_5_kernel method in the following experiments.

### 3.6. Predictive Performance Experiments on an Independent Test Set

To further validate the generalization performance, we conduct the experiments on the independent Strict_data dataset and Nonstrict_data dataset. The ROC curves are shown in Figures 8(a) and 8(b). The AUC value of the BERT-PPII model is 0.827 on the independent Strict_data dataset, and the value is 0.783 on the independent NonStrict_data dataset.

### 3.7. The Comparative Experiments

In this paper, we compare BERT-PPII method with the following methods. To predict PPII helices on a balanced dataset, Siermala et al. [25] employs an artificial neural network (ANN), and Wang et al. [26] adopt a support vector machine (SVM). In contrast, O'Brien KT [30] proposed the PPIIPRED model, and it predicts PPII helix using a bidirectional recurrent neural network (BRNN) on an unbalanced dataset. We conduct the comparative experiments on both the balanced and unbalanced datasets, respectively. The experimental results are shown in Sections 3.7.1 and 3.7.2, respectively.

#### 3.7.1. The Comparative Experiments on a Balanced Dataset

This section conducts the comparative experiments on the balanced dataset and the comparative methods including ANN [25], SVM [26], random forest (RF), K-Nearest Neighbor (KNN), FAD-BERT [19], EECL [10], Adapt_Kcr [40], and BERT4Bitter [20]. All comparative methods use one-hot to encode the amino acid residues. The evaluation metrics are shown in Tables 4 and 5. On the dataset Strict dataset, compared to the best performing support vector machine algorithm (SVM), the BERT-PPII model improved the ACC value by 9.0% and the AUC by 0.4%, as shown in Table 4. On the NonStrict dataset, compared to the best performing support vector machine (SVM), the BERT-PPII model improved the ACC value by 11.5% and the AUC by 0.4%, as shown in Table 5. The BERT-PPII model has the best performance in predicting the PPII helix.

#### 3.7.2. The Comparative Experiments on an Unbalanced Dataset

PPIIPRED model [30] uses a bidirectional recurrent neural network (BRNN) to predict the PPII helix, and we employ PPIIPRED model as the comparative method on the unbalanced dataset. We divide the unbalanced dataset (Strict_data, NonStrict_data) into training set, validation set and test set, and their ratio is 3 : 1 : 1. The experimental result is shown in Table 6 and Figure 9, and its shows that our model outperforms PPIIPRED in predicting the PPII helix. On the Strict_data dataset, the Spec, MCC, and ACC values of the proposed method are 0.99, 0.44, and 0.980, respectively. Compared to the PPIIPRED method, the values of Spec, MCC, and ACC have been improved about 1%, 7%, and 1%, respectively. On the NonStrict_data dataset, the Spec, MCC, and ACC values of the proposed method are 0.99, 0.43, and 0.966, respectively. Compared to the PPIIPRED method, the values of Spec, MCC, and ACC have been improved about 2%, 5% and 1.7%, respectively. The above experiments show that our method can achieve the best performance in predicting the PPII helix structure.

## 4. Conclusions

The PPII helix plays a very important role in many biochemical processes, and it is necessary to quickly and accurately predict the PPII helix. However, it is a time-consuming and expensive work to identify PPII helix using traditional physical and chemical experimental methods. In this study, to some extent, protein sequences also have their own arrangement motifs, which constitute the structure of proteins in space and function in organisms. Due to the protein sequences are similar to the natural language, we can apply the natural language technology to the area of protein sequences. We propose a new model BERT-PPII to identify the PPII helix. The BERT-based BERT-PPII model automatically generates the feature descriptors according to the original amino acid sequence, and it does not need any system design and feature coding selection. We use BERT encoding mechanism to generate the *CLS* vector as the protein sequence feature and fuse it and the CNN local feature vector to enhance feature expression. A large number of experiments have shown that BERT-PPII achieves a better performance than the existing methods. In particular, our method is better than the PPIIPRED on the strict dataset. The ACC value of our method is 1% higher than that of PPIIPRED on the unbalanced datasets. Accuracy (ACC) is 2% higher than PPIIPRED on less stringent datasets. The high prediction performance of our model BERT-PPII enables it to provide robust performance and distinguish between PPII helix and non-PPII helix.

## Figures and Tables

**Figure 1:** The flowchart of BERT-PPII model including input protein sequence samples, BERT embedding encoding and global feature extraction, local feature extraction by multichannel convolution, multifeature fusion, and prediction. It is assumed that the sliding window size is 13 and the amino acid residues in the sample are separated by space in the figure.

**Figure 2:** Some primary sequences of protein sequence (PDB id: 7ODCA) are assigned secondary structure conformations by DSSP algorithm. This graph is derived from the online PPII and secondary structure assignment database developed by Chebrek et al. [35]. In the graph, a letter represents a specific conformation, and its color relates to different secondary structure categories.

**Figure 3:** The Multichannel CNN model.

**Figure 4:** (a) Positive sample; (b) negative sample.

**Figure 5:** The amino acid composition of PPII and Non-PPII.

**Figure 6:** (a) The ROC of BERT-PPII model with different sliding window sizes on the balanced Strict_data test set, WS_9 means that the number of amino acid residues is 9. (b) The ROC plots of BERT-PPII model with different sliding window sizes on the balanced NonStrict_data test set.

**Figure 7:** The ROC plots of the Multichannel CNN model with different integration of n-gram channels on the balanced Strict_data test set.

**Figure 8:** (a) The ROC plot of the BRET-PPII model on the Strict independent test set; (b) The ROC plot of the BERT-PPII model on the NonStrict independent test set. TPR represents the rate that is correctly judged to be positive, and FPR represents the rate that is wrongly judged to be positive.

**Figure 9:** (a) Performance comparison between our algorithm and PPIIPRED on (a) Strict_data dataset and (b) NonStrict_data dataset, respectively.

**Table 1:** The dataset under strict definition (Strict_data).

Dataset	Number of sequence	Number of PPII	Number of non-PPII	Total
Training set	6561	36622	1494487	1531109
Test set	1640	9068	382819	391887
Independent test set	920	4855	201537	206392

**Table 2:** The dataset under less strict definition (NonStrict_data).

Dataset	Number of sequence	Number of PPII	Number of non-PPII	Total
Training set	7121	64490	1554142	1618432
Test set	1781	15880	379276	395156
Independent test set	1001	8639	208785	217424

**Table 3:** The Comparative experiments of the BERT-PPII with different n-gram channel combinations on a balanced Strict_data test set.

Dataset	Window size	Sens	Spec	MCC	ACC
Stirct_data	3_kernel	0.636	0.846	0.491	0.741
	3_4_kernel	0.644	0.847	0.501	0.745
	3_4_5_kernel	0.661	0.841	0.510	0.751
	3_4_5_6_kernel	0.610	0.871	0.498	0.741
	3_4_5_6_7_kernel	0.640	0.854	0.510	0.747

**Table 4:** The comparative experiments on balanced Strict_data dataset.

Methods	Sens	Spec	MCC	ACC	AUC
ANN [25]	0.749	0.736	0.485	0.742	0.742
SVM [26]	0.673	0.841	0.493	0.744	0.822
RF	0.738	0.841	0.554	0.776	0.776
KNN	0.558	0.739	0.302	0.648	0.648
FAD-BERT [19]	0.660	0.821	0.492	0.741	0.752
EECL [10]	0.765	0.776	0.540	0.770	0.770
Adapt_Kcr [40]	0.792	0.767	0.559	0.779	0.855
BERT4Bitter [20]	0.661	0.825	0.493	0.744	0.762
**OUR**	**0.661**	**0.838**	**0.198**	**0.834**	**0.826**

**Table 5:** The comparative experiments on balanced NonStrict_data dataset.

Methods	Sens	Spec	MCC	ACC	AUC
ANN [25]	0.701	0.734	0.435	0.717	0.742
SVM [26]	0.629	0.789	0.423	0.709	0.822
RF	0.681	0.810	0.490	0.746	0.746
KNN	0.636	0.639	0.275	0.637	0.648
FAD-BERT [19]	0.581	0.797	0.411	0.732	0.733
EECL [10]	0.748	0.724	0.472	0.736	0.736
Adapt_Kcr [40]	0.751	0.736	0.487	0.744	0.823
BERT4Bitter [20]	0.590	0.798	0.397	0.695	0.743
**OUR**	**0.559**	**0.833**	**0.219**	**0.824**	**0.826**

**Table 6:** The comparative experiments with on unbalanced Strict_data dataset and NonStrict_data dataset.

Dataset	Methods	Sens	Spec	MCC	ACC
Strict_data	PPIIPRED	0.38	0.98	0.37	0.971
	**OUR**	0.30	0.99	0.44	0.980
NonStrict_data	PPIIPRED	0.43	0.97	0.38	0.949
	**OUR**	**0.30**	**0.99**	**0.43**	**0.966**

## Data Availability

The data that support the findings of this study are openly available at https://github.com/Cambridge-F/BERT-PPII.git.
